The article "The impact of adjacent habitats on population dynamics of red cotton bugs and lint quality" was retracted in 2022. Reasons: compromised peer review; a conflict of interest; concerns about the authorship.

# The impact of adjacent habitats on population dynamics of red cotton bugs and lint quality

**DOI:** 10.1371/journal.pone.0242787

**Published:** 2020-12-31

**Authors:** Haider Karar, Muhammad Amjad Bashir, Khalid Ali Khan, Hamed A. Ghramh, Sagheer Atta, Mohammad Javed Ansari, Zubair Ahmad, Farmanur Rahman Khan

**Affiliations:** 1 Mango Research Institute, Multan, Pakistan; 2 Department of Plant Protection Faculty of Agricultural Sciences, Ghazi University Dera Ghazi Khan Punjab, Punjab, Pakistan; 3 Research Center for Advanced Materials Science (RCAMS), King Khalid University, Abha, Saudi Arabia; 4 Unit of Bee Research and Honey Production, Faculty of Science, King Khalid University, Abha, Saudi Arabia; 5 Biology Department, Faculty of Sciences and Arts, King Khalid University, Dhahran Al Janoub, Saudi Arabia; 6 Department of Botany Hindu College Moradabad, Moradabad, Uttar Pradesh, India; 7 Department of Biology, Deanship of Educational Services, Qassim University, Buraidah, Al Qassim, Saudi Arabia; Harran University, TURKEY

## Abstract

Red cotton bugs [*Dysdercus* spp. (Hemiptera: Pyrrhocoridae] are among the most destructive pests of cotton and many other crops. Red cotton bugs (RCBs hereafter) damage cotton plants by sucking sap and deteriorate lint by staining. The incidence of RCBs causes boll injury along the field margins neighboring with various peripheral areas. The adjacent habitat/crops strongly mediate the population dynamics of RCBs. However, limited is known about the impact of adjacent habitat on population dynamics of RCBs and lint quality. This two-year field study evaluated the impact of adjacent habitat (okra, unpaved road, water channel and *Eucalyptus* trees) on population dynamics of RCBs and lint quality of cotton. The RCBs were sampled weekly from margins to 4 meter inside the cotton field. The RCBs’ populations were monitored and plucked cotton bolls were examined for internal damage. The highest incidence of RCBs was recorded for cotton field adjacent to okra and water channel. Similarly, the highest number of damaged bolls were observed for the field side neighboring with okra and water channel. Furthermore, the highest number of unopened bolls were recorded for okra and water channel sides with higher percentage of yellowish lint. Field sides bordering with *Eucalyptus* trees and unpaved road had lower RCBs incidence and lint staining. Nonetheless, RCBs incidence was higher at field margins compared to field center indicating that population was strongly affected by adjacent habitat. It is concluded that sowing okra and weedy water channels adjacent to cotton would support RCBs population and subsequent lint staining. Therefore, water channels must be kept weed-free and okra should not be sown adjacent to cotton. Nonetheless, detailed studies are needed to compute monetary damages caused by cotton pests to the crop. Furthermore, effective management strategies must be developed to manage RCBs in cotton to avoid lint-staining problem.

## Introduction

Cotton (*Gossypium hirsutum* L.) is among the most important cash crops grown globally and natural fiber obtained from the crop is used in textile industry [1]. Cotton is called ‘white gold’ and plays a vital role in strengthening the economies of countries like Pakistan. Cotton contributes 68% towards foreign exchange [2] and 62.3% of total exports in Pakistan [3]. Several insects and diseases infest cotton crop, which exert severe quality and quantity losses. Red cotton bugs’ (RCBs) infestation in Pakistan not only decreases market price of cotton but also produces low quality seed [4]. Cotton bugs have become economically important pests in several regions of the world [5]. The continuing changes in production practices are resulting in the outbreak of new pests.

The boll-feeding cotton bugs include several species of bugs and stinkbugs. Green stinkbug [*Acrosternum hilare* (Say)], brown stinkbug [*Euschistus servus* (Say)] and southern green stinkbug (*Nezara viridula* L.) are the most dominant pests in southern America [6]. These pests together with other insects cause significant reduction in yield and lint quality. These insects feed on developing bolls and deform them, lower yield and quality, and cause boll abscission [7–14]. Stinkbugs’ feeding also ensures microorganisms’ entry to the fruits, resulting in physiological damage and fruit degradation [15–20]. The peak yield losses in South Carolina due to stinkbugs were recorded during 2005 [21].

The RCBs are the most destructive cotton pests because of their impact on lint staining [22, 23]. These bugs feed on emerging bolls and mature seeds, and transmit cotton staining fungi (*Nematospora gossypii*), which develops on lint and seed [24, 25]. Furthermore, the fungal pathogen transmitted during feeding causes reddening of cotton lint [26]. The RCBs cause serious damage by feeding with their strong piercing/sucking mouthparts. Nymphs and adults feed on bolls and ripened seeds [27]. These bugs are not only serious pests of cotton, but also infest several other crops, including okra, hollyhock and hibiscus [28]. The bugs were ignored for a long duration due to their minor losses. However, this ignorance has led to the outbreak of the bugs as serious pest resulting in low crop yield [29].

The RCBs stain the lint [30], and negatively affect seed weight, oil contents and seed viability [31]. Several or only a few seeds within each lock may be affected [32]. The RCBs are also sap sucking insect pests of okra. They did not reduce the yield significantly, but lower fruit quality by inflicting a rusty appearance on the surface [33]. Furthermore, these are also severe pests of other economically important plants such as legumes, red gram [34] and Portia tree [35].

Several studies have indicated that adjacent habitat affects population dynamics of RCBs. However, there is lack of information regarding the impact of peripheral areas and climatic factors on population dynamics of RCBs. Many studies have addressed the dispersal and movement of stinkbugs within and between different crops and habitats [36–41]. However, numerous questions remain unanswered about the influence of adjacent agronomic crops and wild hosts on the movement and development of RCBs along the margins of cotton fields. To address these critical questions, current study was planned to infer the impact of peripheral areas of population dynamics of RCBs. Furthermore, inferring the impact of RCBs on quality and quantity of cotton was the second objective of the study.

## Materials and methods

This two-year field study was conducted at a Government Agricultural Farm near Vegetable Research Sub Station, Multan during 2011–12 and 2012–13. The study required no specific permissions as the farm is devoted for cotton and other field crops’ research and no endangered or protected species were involved. Cotton crop was sown on 7^th^ and 15^th^ May during 2012 and 2013, respectively. The experimental field was surrounded by four different peripheral areas on each side. The field was surrounded by okra crop, weedy water channel, unpaved road and *Eucalyptus* trees. Four rows of cotton plants on each side were selected to monitor the population dynamics of RCB and lint. The sampling for RCBs was done on weekly basis from 30 days after sowing until harvest. One hundred and fifty unopened bolls were plucked and observed. The center of the field was regarded as control for comparison. Bolls were plucked in October from the border of each peripheral area. The bolls were kept in paper bags for seven days in a hot and cool chamber. The bolls were dissected and the condition of the lint was observed. There was no control on the other insect pests, which may be treated as a limitation of the study. However, cotton staining is caused by RCBs and we were interested to know whether lint quality is influenced by RCBs. Weather data of both seasons is summarized in Fig 1.

**Fig 1:** Climatic data of the experimental site during cotton growing seasons of 2012 and 2013.

### Data collection

The population of RCBs was recorded from 10 randomly selected plants per row and averaged. The number of unopened bolls were counted carefully form 50 randomly selected plants on each side of the field and averaged for each side, separately. The locks of bolls were opened with sharp knife and yellowish and whitish lint was noted. The percentage of yellowish and whitish color was then calculated.

### Statistical analysis

The collected data were analyzed according to Fisher’s Analysis of variance technique (ANOVA). One-way ANOVA was used to test the significance in data. Significant differences were noted among experimental years. Therefore, data of each year was analyzed and presented separately. The data were analyzed on Statistix version 9 (www.statistix.com/freetrial.html) (Lawes Agricultural Trust Rothamsted Experimental Station, Rothamsted, UK). The means were separated by Tukey’s honestly significant difference test at 5% probability where ANOVA indicated significant differences.

## Results

**S**ignificant differences were noted among various peripheral areas for number of unopened bolls during 2012 (Table 1). Field side adjacent to okra crop observed the highest number of unopened cotton bolls per plant followed by weedy water channel during 2012. The lowest number of unopened bolls were recorded for the field side adjacent to *Eucalyptus* tree during 2012 (Table 2). Similar to 2012, peripheral areas significantly differed (Table 1) for number of unopened bolls during 2013. Okra side had the highest number of unopened cotton bolls followed by weedy water channel during 2012. All other peripheral sides had no unopened bolls during 2012 (Table 2).

**Table 1:** Analysis of variance of red cotton bugs infestation, number of unopened bolls and lint staining during 2012 and 2013.

Source	Degree of freedom	Sum of squares	Mean squares	F value	P value
**2012**					
**Unopened bolls plant**^**-1**^					
Habitat	4	1106.98	276.74	217.38	< 0.0001*
Error	10	12.73	1.27		
**RCBs plant**^**-1**^					
Habitat	4	936.13	234.03	75.93	< 0.0001*
Error	10	30.82	3.08		
**Yellowish lint (%)**					
Habitat	4	1871.61	467.90	85.84	< 0.0001*
Error	10	54.51	5.45		
**Whitish Lint (%)**					
Habitat	4	1871.61	467.90	141.52	< 0.0001*
Error	10	33.06	3.31		
**2013**					
**Unopened bolls plant**^**-1**^					
Habitat	4	0.63	0.16	285.87	< 0.0001*
Error	10	0.01	0.00		
**RCBs plant**^**-1**^					
Habitat	4	10.31	2.58	135.04	< 0.0001*
Error	10	0.19	0.02		
**Yellowish lint (%)**					
Habitat	4	5.25	1.31	27.21	< 0.0001*
Error	10	0.48	0.05		
**Whitish Lint (%)**					
Habitat	4	4.95	1.24	1.61	0.25NS
Error	10	7.67	0.77		

* = significant, NS = non-significant

**Table 2:** The impact of different peripheral areas on red cotton bugs population, number of unopened bolls and lint quality of cotton during 2012 and 2013.

Habitat	Unopened bolls plant^-1^	RCBs plant^-1^	Yellowish lint (%)	Whitish Lint (%)
**2012**				
**Unpaved road**	7.55 cd	18.30 c	63.73 b	36.27 a
**Water channel**	20.30 b	25.15 a	87.96 a	12.04 c
**Okra crop**	26.60 a	27.05 a	91.43 a	8.57 c
***Eucalyptus* Trees**	3.75 d	4.55 d	69.07 b	30.93 b
**Control**	8.95 c	18.10 b	69.32 b	30.68 b
**HSD 5%**	4.77	5.52	10.41	4.88
**F value**	178.52	69.48	68.93	113.55
**2013**				
**Unpaved road**	0.00 c	9.30 c	0.00 b	100
**Water channel**	0.07 b	15.15 b	1.18 a	98.89
**Okra crop**	0.52 a	21.05 a	1.23 a	98.77
**Eucalyptus Trees**	0.00 c	2.27 d	0.00 b	100
**Control**	0.00 c	12.31 b	0.00 b	100
**HSD 5%**	0.07	2.95	0.65	2.73
**F value**	278.24	132.31	24.36	NS

Means sharing similar letters are not significantly different by Tukey HSD at P = 0.05 HSD = Honestly significant difference value

**S**ignificant differences were noted among various peripheral areas regarding the population of RCBs during both years (Table 1). Okra side recorded the highest RCBs’ infestation during both years, which was statistically similar to weedy water channel. The RCBs population on unpaved road side and control treatment was similar. *Eucalyptus* tree side recorded the lowest RCB population during each year (Table 2).

**S**ignificant differences were observed between various peripheral areas regarding the percentage of yellowish lint (Table 1). The okra and water channel sides had significantly higher percentage of yellowish lint compared with other sides. Control treatment *Eucalyptus* trees and unpaved road had statistically similar percentage of yellowish lint during 2012 (Table 2). A very low percentage of yellowish lint was recorded during 2013 with significant differences (Table 1) among peripheral areas. The okra and water channel sides had higher percentages of yellowish lint compared to the rest of the peripheral areas.

Various peripheral areas significantly differed for whitish lint percentage during 2012 (Table 1). Unpaved road side had greater percentage of whitish lint, which was statistically similar to *Eucalyptus* tree side and control treatment. Water channel and okra sides had statistically less whitish lint during 2012 (Table 2). Statistically similar results were observed for whitish lint for all peripheral areas during 2013 (Table 1).

During 2012 and 2013 okra side has a greater population of RCBs with more yellowish lint. Similarly, *Eucalyptus* tree side and control treatment had low population with less yellowish lint during both years (Fig 2).

**Fig 2:** Average population of red cotton bugs and their impact on lint quality during 2012 and 2013. YL = yellowish lint, WL = whitish lint; RCB = red cotton bugs; UOB = unopened bolls.

## Discussion

The results of the current study suggested that RCBs emigrate from surrounding habitats where they reproduce and feed on developing bolls. Several studies have indicated that control of stinkbugs is critical in cotton sown adjacent to soybean [42] and peanut [43–45] than other crops [46–48]. Higher population of RCBs was noted near field margins than field center. From cultural control point of view, this data suggests that cotton should be isolated to possible extent possible from other crops, which may harbor these bugs. Row orientation can affect RCBs movement [49, 50] and oviposition. The strong effect of field border in the current study is in line with the earlier studies [51]. Trap crops can be useful to minimize RCBs movement between crop rows. Intensive management practices should be opted to managed RCBs where adjacent areas are sown with crops harboring these bugs.

Bolls are affected by RCBs during boll development phase [52, 53]. Therefore, crop is at risk during early season [54]. However, crops with early maturity could act as potential traps for RCBs [55–57].

Sorghum has the potential to act as trap crop for RCBs emerging from maize and groundnut and infesting cotton. Fewer insecticides are required to control RCBs if sorghum is sown as trap crop [58]. Trap crops, fallow and natural areas along cotton field margins can add significant contribution towards biological control of RCBs by increased movement of predators in cotton and enhance action of natural enemies [59–61].

Our results suggested that more numbers of unopened cotton bolls were recorded during 2012 than 2013 with higher percentage of yellowish cotton on okra side and weedy water channels. Similarly, less yellowish cotton was observed during 2013. There were significant differences for RCBs’ population per plants during both years indicating that weather factors play a pivotal role in population dynamics of RCBs and lint staining. Weather factors played a major role during 2012 where 91% of lint become yellow because of more rainfall and high relative humidity. The okra sider observed the highest population of RCBs during both years of the study. The reason is that okra is the most susceptible host of RCBs and cotton crop parallel to okra was more affected than rest of the peripheral areas. The results are inconformity with Reeves et al. [62] who reported that adjacent habitat has significant impact on RCBs.

Weedy water channel acts as a hibernating and breeding place and identified as a second highest percentage of yellowish cotton. The insects breed and spread to all cotton field from these two places as most of the young pests continue spreading into the fields. On the other hand, unpaved road and tree sides have less unopened bolls and yellowish lint percentage. The reasons behind this could be that both these areas adjacent to cotton and do not have cracks and hibernating places, so less number of unopened bolls and a lesser percentage of yellowish lint was recorded. Cotton discoloration is undesirable in the textile mill because the lint surface is deteriorated. Deterioration of the lint surface increases its roughness and affects the way the fibers slide across each other during the spinning process. Field weathered cotton suffers increased fiber breakage resulting in higher short fiber content, which lowers the yam evenness and quality [63].

## Conclusion

The population of red cotton bugs was significantly altered by adjacent habitats and the highest negative impacts were posed by okra and weedy water channel sides. Both habitats resulted in more yellowish lint than other habitats. To produce whitish lint, the red cotton bugs should be controlled by keeping water channels clean and avoid sowing of okra near cotton crop.
